# Image Features of Dynamic Enhanced Computed Tomography Scanning Combined with Digestive Endoscopy in the Treatment of Gastroesophageal Varices and Nursing of Esophagogastric Gastric Varices Bleeding

**DOI:** 10.1155/2022/7926114

**Published:** 2022-06-20

**Authors:** Huijun Ding

**Affiliations:** Endoscopy Center, Lin'an First People's Hospital, Lin'an, Hangzhou, 311300 Zhejiang, China

## Abstract

The objective of this study was to investigate the application of dynamic contrast-enhanced CT images in the nursing of patients with gastroesophageal varices (GOV) treated by digestive endoscopy and its role in relieving bleeding symptoms. A total of 60 patients with liver cirrhosis and GOV were selected as the research objects. According to whether CT was used to evaluate the position of tissue adhesion embolism, the patients were divided into the control group (24 cases) and the observation group (36 cases). The treatment effect and bleeding situation of patients in the two groups were analyzed and compared. The results showed that the main portal vein pressure (17.24 ± 1.02 cmH_2_O), liver function recovery effect (2.84 ± 0.45 points), and total effective rate (100%) in observation group were better than those in control group (9.70 ± 1.22 cmH_2_O, 0.95 ± 0.72 points, and 79.17%, respectively) (*P* < 0.05). In addition, the bleeding rate in observation group (0%) was significantly lower than that in control group (16.67%) (*P* < 0.05). In conclusion, dynamically enhanced CT scan images combined with digestive endoscopy can help improve the therapeutic effect of GOV and reduce postoperative bleeding, which was worthy of clinical application and promotion.

## 1. Introduction

Cirrhosis is one of the common chronic diseases in gastroenterology, and gastroesophageal varices (GOV) is one of its common complications, with an incidence of more than 50% [1]. GOV is prone to esophageal vein rupture and bleeding, and clinical studies have shown that patients with cirrhosis-GOV have about 25% bleeding probability within 2 years [2]. Esophagogastric gastric varices bleeding (EGVB) is fairly serious [3]. Once EGVB occurs, it can lead to repeated bleeding, which has a high mortality and disability rate for patients and is one of the main causes of death for patients [4, 5]. Therefore, how to accurately treat GOV to prevent the occurrence of EGVB is of great significance to patients with cirrhosis.

At the present stage, the clinical treatment of GOV is embolization of the varicose vein in the fundus of the stomach and occlusion of the varicose pathway. The treatment methods include drug therapy, digestive endoscopy, and surgical procedure, among which the digestive endoscopy is recognized by clinical patients due to its minimally invasive procedure [6]. In addition, with the rapid development and popularity of the technique of digestive endoscopy, the treatment and prevention of EGVB under the condition of digestive endoscopy have become the first-line therapy [7]. The specific surgical procedures for the treatment using digestive endoscopy are loop ligature and tissue glue injection of esophageal varices [8]. In the course of treatment using digestive endoscopy, the treatment effect is influenced by whether the tissue adhesives could embolize the starting vein accurately [9]. Evaluation of the location of embolism is an issue that needs to be considered to provide timely and effective postoperative care.

The standard of GOV is gastroscopy, but this method is invasive and may induce bleeding with many restrictive factors [7]. With the maturity of imaging technology, multislice spiral CT has been widely applied in vascular examination, such as computed tomography (CT) portal venography (CTPV) [10]. However, CTPV is expensive and cannot be widely used in clinical practice due to the complexity of the operation and restricted conventional scanning image resolution. To solve the complicated operation, unpopularity in clinic, and clarity of image, some experts propose that three dimensional slicer (3D slicer) software could be used to reconstruct the blood vessels in the portal vein system of upper abdomen during the CT dynamic enhanced scanning, so as to improve the application value of images [11].

Therefore, in this study, the 3D slice software was used to reconstruct the position of dynamic enhanced CT scan images of tissue adhesion embolism, and the conditions of patients with GOV were evaluated by using the gastrointestinal endoscopy to assist the nursing work of patients with GOV. By evaluating the therapeutic effect and postoperative bleeding of patients before and after treatment, the application value of CT combined with digestive endoscopy was evaluated. This study was aimed at providing reference value for improving the treatment effect of patients with GOV and bleeding and elevating the survival rate of patients.

## 2. Research Methods

### 2.1. Research Subjects

In this study, 60 patients with cirrhosis complicated with gastric varices in the hospital from June 2019 to June 2021 were selected as the subjects. There were 39 male patients and 21 female patients, ranging in age from 20 to 80 years old, with an average age of 51.32 ± 7.22 years old. According to the results of liver function grading [12], there were 14 cases of grade A, 20 cases of grade B, and 26 cases of grade C. The patients were divided into a control group and an observation group according to whether CT dynamic scanning was used to monitor the location of tissue adhesive embolization during treatment. 24 cases in the control group were treated with loop ligature+tissue glue injection only under digestive endoscopy. In the observation group, 36 cases were examined by dynamic contrast-enhanced CT scan images combined with digestive endoscopy. Treatment effect and bleeding of the two groups were analyzed and compared. The study had been approved by ethics committee of hospital. The patients and their families signed the informed consent forms.

Inclusion criteria were as follows: (a) all patients suffered from alcoholic cirrhosis; (b) the patients signed the informed consents and voluntarily participated in the experiment; (c) all patients were over 18 years old; (d) all the patients were diagnosed as GOV by magnetic resonance imaging (MRI), CT, gastroscopy, and other examinations according to *Standard Trial Plan of Endoscopic Diagnosis and Treatment of Esophageal and Gastric Varices* [13], and (e) none of the patients had bleeding symptoms.

Exclusion criteria were as follows: (a) patients with serious organ dysfunction such as heart and kidney, cancer, systemic infectious diseases, abnormal immune system, or blood tests; (b) patients with unclear mental awareness; (c) patients who were unwilling to cooperate during treatment; (d) pregnant women; (e) patients who had previously received relevant surgical treatment; and (f) patients with contraindications for treatment.

### 2.2. CT Examination Method

64-slice spiral CT scanner was performed. Before the examination, the patient should fast for more than 6 hours and take oral water (500 mL) to fill the digestive tract 15 minutes before the examination. An indwelling needle was placed in a vein in the forearm at the same time. In addition, the scanning process is needed to be performed after inhaling and holding the breath, so the patient's breathing had to be contacted before the examination to facilitate the smooth operation of the examination. The patient was placed in supine position and scanned the area of the abdomen from the top of the diaphragm to the level of the iliac crest. First, a horizontal upper abdominal CT scan was required to determine the site of the disease. Then, a double-barbed high-pressure syringe was used to inject 80-100 mL of nonionic contrast agent iodihydrin (3.0 mL/s) through indwelling needle, and dynamic enhanced scanning was performed in arterial phase (20 s), portal vein phase (60 s), and equilibrium phase (120 s). The scanning parameters were as follows: tube voltage was 120 kV, tube current was 240 mA, layer thickness was 5 mm, pitch was 0.983, field of view was 36 cm, matrix was 510 × 510, and the duration was 0.7 s.

### 2.3. Treatment Way

All the patients were treated with loop ligature+tissue glue injection under digestive endoscopy, and the patients were ordered to refrain from drinking for at least 8 hours before surgery. Before surgery, anesthesia was required, and then, the distal end of the varicose vein was induced by negative pressure into the transparent cap until the phenomenon of “red vision” appeared. Then, the root of the varicose vein was ligation with loop ligature ring, and the purple color of loop ligature vein was regarded as success. After that, the sandwich method, i.e., “lauromacrogol-tissue glue-laurogol,” was used for tissue glue injection intervention (the lauromacrogol was injected into the injection pipeline to block, then the tissue glue (appropriate amount) was injected into the position of the varicose, and finally the lauromacrogol was injected again to ensure that all tissue glue entered the position of the varicose). The patients in control group received follow-up treatment based on clinical manifestations, and those in the observation group received follow-up treatment based on CT image observation of tissue glue.

### 2.4. Observation Indicators

Main portal vein pressure and liver function score (Child-Pugh) of 2 groups were examined before treatment and 3 months after treatment. GOV recovery efficiency was compared between the two groups (markedly effective: disappeared varices and no bleeding; effective: relieved varicosity, no bleeding; and ineffective or aggravated: no change in varicose, even rupture bleeding). At the same time, the rupture and bleeding of the two groups of patients were compared. Child-Pugh scoring criteria were as follows: the severity of five aspects, such as serum bilirubin level, ascites, and prothrombin time, was scored. Each item could be marked 1~3 points according to the severity, so there were a total of 15 points: 5~6 points: grade A, 7~9 points: grade B, and 10~15 points: grade C.

### 2.5. Statistical Methods

SPSS 22.0 statistical software was used for data processing in this study. The quantity was expressed as *X* ± *S*, *t* test was used, and the number was expressed as %. The statistically significant difference was tested with *χ*^2^, and the standard of statistical significance was *P* < 0.05.

## 3. Results

### 3.1. Comparison on General Data

Figure 1 shows the statistical distribution of the general clinical data of patients in the two groups, such as gender, age, and liver function grade. According to Figure 1, there were no significant differences in gender distribution, age distribution, and liver function distribution between the two groups (*P* > 0.05), which suggested that this study was feasible.

### 3.2. Main Portal Vein Pressure and Child-Pugh Score

Main portal vein pressure and Child-Pugh score of patients in the two groups were statistically compared before and 3 months after treatment, as shown in Table 1. The main portal vein pressure in control group was 38.73 ± 2.97 cmH_2_O before treatment and 29.03 ± 1.77 cmH_2_O after 3 months of treatment. In the observation group, it was 38.91 ± 2.44 cmH_2_O before treatment and 21.83 ± 1.52 cmH_2_O 3 months after treatment. There was no significant difference in main portal vein pressure between the two groups before treatment (*P* < 0.05), and it in both groups decreased 3 months after treatment. However, the degree of reduction in observation group (17.24 ± 1.02 cmH_2_O) was significantly higher than that in control group (9.70 ± 1.22 cmH_2_O) (*P* < 0.05), as shown in Figure 2. The Child-Pugh score of control group was 10.66 ± 1.24 before treatment and 9.78 ± 1.45 after 3 months of treatment; in the observation group, the score was 10.49 ± 1.53 before treatment and 7.94 ± 1.83 after 3 months of treatment. It demonstrated that there was no significant difference in Child-Pugh score between the two groups before treatment (*P* < 0.05), and the reduction of the observation group (2.84 ± 0.45) was significantly higher than that of the control group (0.95 ± 0.72) after 3 months of treatment (*P* < 0.05), as shown in Figure 2.

### 3.3. Total Effective Rate

After statistics, there were 32 cases with markedly effective, 4 cases of effective patients, and 0 cases of ineffective or aggravated patients in the observation group of patients, so the total effective rate was 100%. In the control group, 13 patients were markedly effective, 6 patients were effective, and 5 patients were ineffective or aggravated, so the total effective rate was 79.17%. After comparison, it was found that the total effective rate of the observation group was higher than that of the control group (*P* < 0.05), as shown in Figure 3.

### 3.4. Comparison on Bleeding Rate

Figure 4 shows the comparison of GOV bleeding rate between the two groups after treatment. It was known from the figure that there were no ruptured bleeding patients in the observation group, and 4 of the 5 ineffective or aggravated patients in the control group had ruptured bleeding symptoms. After calculation, the bleeding rate of the control group was 16.67%, and that of the observation group was 0, so the bleeding rate of the observation group was significantly lower than that of the control group (*P* < 0.05). CT images in Figure 4 were posttreatment bleeding examination images of patients in the control group, and splenomegaly existed in 2 patients.

## 4. Discussion

With the increasing incidence of cirrhosis and other liver diseases in clinical practice, the incidence of GOV complications also increases, and rupture and bleeding in severe cases can bring certain life risks to patients [14]. Therefore, timely and effective treatment and alleviation of varices can improve GOV rupture and hemorrhage to a certain extent. At present, the commonly used clinical treatment methods are loop ligature under digestive endoscopy and tissue gel injection. To improve the therapeutic effect using digestive endoscopy, dynamic enhanced CT scanning image-assisted digestive endoscopy was used to ensure the accurate location of tissue glue.

On this basis, loop ligature and tissue glue injection under CT image-assisted digestive endoscopy were used to treat patients with GOV. A number of studies show that loop ligature and tissue glue injection therapy under digestive endoscopy could effectively and significantly improve the portal vein pressure and liver function of patients [15, 16]. In this study, the main portal vein pressure and Child-Pugh score of patients in the control group and the observation group decreased greatly before and 3 months after treatment, which was consistent with the above research results. In addition, the effects of treatment were compared with those with digestive endoscopy alone. The results showed that the main portal vein pressure, liver function recovery effect, and total effective rate of patients in the observation group were better than those in the control group. It is suggested that CT image function could improve the therapeutic effect of digestive endoscopy. Q. Li et al. [17] and Zhu et al. [18] also proposed in their studies that CT images can be used for effective diagnosis and adjuvant treatment of GOV. Zhu et al. [19] also proposed that CT imaging could effectively screen and evaluate the treatment of digestive endoscopy. The results of this study also showed that the bleeding rate (0%) in the observation group was significantly lower than that in the control group (16.67%) (*P* < 0.05). It indicates that using dynamic enhanced CT scanning images to assist in the evaluation of tissue glue embolization to determine the origin of varicose veins can not only improve the treatment effect but also reduce the possibility of postoperative EGVB. Such results are consistent with the research results of Wan et al. [20]. Alessio et al. [21] also proposed that dynamic contrast-enhanced CT scans were helpful in assessing vascular status. They all provide research support for the results of this study.

## 5. Conclusion

In conclusion, dynamic contrast-enhanced CT scan images combined with digestive endoscopy can help improve the nursing effect of patients with GOV and bleeding and reduce the probability of postoperative bleeding, which was worthy of clinical application and promotion. This study showed that image-assisted surgery was an effective method for the treatment of certain clinical diseases, showing good application prospects. However, the number of patients in each group in this study was relatively small, so the accuracy of the findings would have some impact, and further research support was needed.

## Figures and Tables

**Figure 1:** Comparison on general data of patients.

**Figure 2:** Comparison on changes before and after treatment. ^∗^Compared with the control group, *P* < 0.05.

**Figure 3:** Comparison on treatment effect. ^∗^Compared with the control group, *P* < 0.05.

**Figure 4:** Comparison on bleeding rate of patients in two groups. ^∗^Compared with the control group, *P* < 0.05.

**Table 1:** Statistical results of main portal vein pressure and Child-Pugh score of patients.

Indicator		Control group (*n* = 24)	Observation group (*n* = 36)	*t*	*P*
Main portal vein pressure (cmH_2_O)	Before treatment	38.73 ± 2.97	38.91 ± 2.44	1.212	0.121
	3 months after treatment	29.03 ± 1.77	21.83 ± 1.52	16.211	0.001
Child-Pugh score (points)	Before treatment	10.66 ± 1.24	10.49 ± 1.53	1.093	0.508
	3 months after treatment	9.78 ± 1.45	7.94 ± 1.83	12.171	0.012

## Data Availability

The data used to support the findings of this study are available from the corresponding author upon request.
